# Modeling the Temperature Field of the Microwave Heating Asphalt Mixture with the Utilization of a Mathematical Model

**DOI:** 10.1155/2022/9356893

**Published:** 2022-06-29

**Authors:** Yifei Zhang, Qingxian Wang, Bofu Guo

**Affiliations:** ^1^National Engineering Research Center for Highway Maintenance Equipment, Chang'an University, Xi'an 710064, China; ^2^Jiangsu JITRI Road Engineering Technology and Equipment Research Institute Co., Ltd., Xuzhou 221001, China

## Abstract

Microwave heating asphalt mixture is an auspicious method since it requires a minimum level of outside intervention. It has been a recent method with some certain advantages over conventional ones. To obtain the temperature field of microwave heating asphalt mixture utilizing an oblique horn antenna, the aperture field of the oblique horn antenna was deduced based on the Maxwell equations. The three-dimensional mathematical model of a microwave heating asphalt mixture was established by introducing a position relation of the horn caliber called an oblique horn antenna, and the calculation results were simplified and verified by experiments. The results showed that the calculated values of the mathematical model tally with the experimental outcomes. The model is found to be accurate and reliable.

## 1. Introduction

With ever-increasing road mileage around the globe, the focus of pavement construction has shifted from new pavement construction to pavement maintenance and rehabilitation [1, 2]. When compared with methods of conventional asphalt pavement heating such as hot air and infrared, microwave heating has the advantages of less pollution, large penetration into the depths, a small temperature gradient, no thermal inertia, and 100% recycling capability of an old asphalt mixture [3, 4]. Thus, microwave heat time (cycles) has a limited influence on asphalt aging within a controlled temperature range [5], with no air emissions or liquid pollutants [6]. Moreover, microwave heating can ensure rapid, uniform, and deep penetration [7].

The amount of electricity used by microwave devices is much less than those required to produce a similar effect by electromagnetic induction [8]. Therefore, microwave heating has been a more and more widely employed technique in the maintenance of asphalt roads. The widely benefitted features of this method can be found in [6, 9, 10].

The device used for mixing microwaved heated asphalt is mainly composed of a magnetron, a power supply, a horn antenna, and a cooling device. The size of the horn antenna is closely related to microwave frequency. To reduce the volume of microwave heating equipment and improve the microwave power density per unit area of an asphalt road, an oblique horn antenna is utilized in microwave maintenance equipment in practical implementations. The scholars in [11–17] researched the aperture field of the straight horn antenna according to the Maxwell equations. The propagation direction of the microwave is perpendicular to the aperture of the horn, and the microwave power is the largest at the center of the aperture of the horn antenna. Thus, the mathematical models of the temperature field are established based on the above aperture field. While the highest temperature is located directly below the horn antenna, the highest temperature is located below the center of the horn antenna at the same depth. However, it is found that the high-temperature area after heating with the oblique horn antenna is not located at the center of the horn aperture but deviates to the bevel direction of the horn antenna; in other words, the aperture field of the oblique horn antenna is found to be different from that of the straight horn antenna and cannot be replaced by the aperture field of the straight horn antenna. Therefore, more research is needed to be conducted in this direction.

## 2. The Aperture Field of an Oblique Horn Antenna Port

The straight horn antenna and oblique horn antenna are shown in Figure 1 [18, 19]. The magnetron is installed on the side of the straight horn antenna. Because the magnetron size is large, it can only be placed after increasing the height of the horn antenna and the size of the bell aperture or increasing the distance between adjacent horn antennas is necessary, which will inevitably lead to a lower power density and slower heating. While the magnetron is installed on the top of the oblique horn antenna with a compact structure and a lower height, the adjacent horn antennas can be contacted. The density of the output power of the horn is larger and so is higher the heating efficiency.

In the oblique horn antenna shown in Figure 2, a straight horn antenna is constructed by extending the oblique edge M'm and right angle NF to intersect at point O, and the included angle is *β*. The angle bisector of *β* and the antenna bottom edge M'n intersect at the O” point, and the vertical line NO' is made from the point N and extended, which is compared with the oblique edge at the point M. The constructed △OMN is the standard H-plane horn antenna, and the microwave can be considered to be transmitted from point O and propagated along the direction of OO'.

Equation (1) presents the well-known electromagnetic field equations where $\overset{⟶}{E}$ denotes electric field, $\overset{⟶}{H}$ represents magnetic intensity, ∇ notation and ∇x notation denote gradient and curl operations, respectively, *j* denotes the total current per unit area, *ρ* denotes the total charge per unit area, and *μ* and *ε* denote the spaces related to permittable and permeable.

(1) $$\begin{array}{c} \begin{array}{c} \nabla \times \overset{⟶}{E}=-j\omega \mu \overset{⟶}{H},\\ \nabla \times \overset{⟶}{H}=j\omega \varepsilon \overset{⟶}{E}. \end{array} \end{array}$$

Then, the cylindrical form, *H*_*y*_, *H*_*φ*_, *H*_*ρ*_ and *E*_*y*_, *E*_*φ*_, *E*_*ρ*_, of this equation is rewritten by

(2) $$\begin{array}{c} \begin{array}{c} \left.\begin{array}{c} \frac{1}{\rho }\frac{\partial \left(\rho E_{\phi }\right)}{\partial \rho }-\frac{1}{\rho }\frac{\partial E_{\rho }}{\partial \phi }=-j\omega \mu H_{y}\\ \frac{1}{\rho }\frac{\partial E_{y}}{\partial \phi }-\frac{\partial E_{\phi }}{\partial y}=-j\omega \mu H_{\rho }\\ \frac{\partial E_{\rho }}{\partial y}-\frac{\partial E_{y}}{\partial \rho }=-j\omega \mu H_{\phi } \end{array}\right\},\\ \left.\begin{array}{c} \frac{1}{\rho }\frac{\partial \left(\rho H_{\phi }\right)}{\partial \rho }-\frac{1}{\rho }\frac{\partial H_{\rho }}{\partial \phi }=j\omega \varepsilon E_{y}\\ \frac{1}{\rho }\frac{\partial H_{y}}{\partial \phi }-\frac{\partial H_{\phi }}{\partial y}=j\omega \varepsilon E_{\rho }\\ \frac{\partial H_{\rho }}{\partial y}-\frac{\partial H_{y}}{\partial \rho }=j\omega \varepsilon E_{\phi } \end{array}\right\}. \end{array} \end{array}$$

Under the single-mode excitation of the TE_10_ wave, the expression of the field quantity in the H-plane sector horn can be obtained by resolving the above equation system. Thus,

(3) $$\begin{array}{c} \left.\begin{array}{c} E_{y}=C\cos n\phi H_{n}^{\left(2\right)}\left(k\rho \right)\\ H_{\phi }=-j\frac{k}{{\omega \mu }_{0}}C\cos n\phi \frac{d}{d\left(k\rho \right)}H_{n}^{\left(2\right)}\left(k\rho \right)\\ H_{\rho }=-j\frac{n}{{\omega \mu }_{0}\rho }C\sin n\phi H_{n}^{\left(2\right)}\left(k\rho \right) \end{array}\right\}, \end{array}$$

where *n* = *π*/2*φ*_*H*_ and $k=\omega \sqrt{\mu_{0}\varepsilon_{0}}$. *H*_*n*_^(2)^(*kρ*) is called the second kind of the Hankel function with (*kρ*) the number of cases, which represents the outward wave propagating from the top of the horn. When the value (*kρ*) grows large, the Hankel function has the following asymptotic formula expressed by

(4) $$\begin{array}{c} \begin{array}{c} H_{n}^{\left(2\right)}\left(k\rho \right)=\sqrt{\frac{2}{\pi k\rho }}e^{-j\left(kp-\left(\left(2n+1\right)/4\right)\pi \right)}. \end{array} \end{array}$$

Far away from the top of the horn, the *H*_*ρ*_ is much smaller than the *H*_*φ*_ and can be ignored. Therefore, there exist only two electromagnetic field components, namely, *E*_*y*_ and *H*_*φ*_. Thus,

(5) $$\begin{array}{c} \left.\begin{array}{c} E_{y}=C\sqrt{\frac{2}{\pi k\rho }}\cos n\phi e^{-j\left[k\rho -\left(n+\left(1/2\right)\right)\left(\pi /2\right)\right]}\\ H_{\phi }=-\frac{E_{y}}{120\pi }\\ H_{\rho }=H_{y}=E_{\phi }=E_{\rho }=0 \end{array}\right\}. \end{array}$$

Suppose that the amplitude of the electric field is cosine distributed along the *Y* direction, according to cos*nϕ* = cos(*π*/2)(*ϕ*/*ϕ*_*H*_), where *φ*_*H*_ is the half of the opening angle of the H-plane fan-shaped horn. Namely,

(6) $$\begin{array}{c} \begin{array}{c} \phi_{H}=\tan^{-1}\left(\frac{D_{1}/2}{L_{H}}\right)\approx \frac{D_{1}}{2L_{H}},\\ \phi =\tan^{-1}\left(\frac{X_{S}}{L_{H}}\right)\approx \frac{X_{S}}{L_{H}}. \end{array} \end{array}$$

Therefore, cos*nϕ* = cos(*πX*_*S*_/*D*_1_).

Besides, Equation (1) can be expressed in the form of cylindrical coordinates shown in Figure 3.

In addition, the phase of each point of the aperture field is different according to the characteristics of surface waves. Figure 3 depicts that *X*_*S*_ is away from the midpoint O of the aperture at point M, and the phase of the field lags the phase at the center point O, which is caused by the travel difference.

(7) $$\begin{array}{c} \text{MN}=\sqrt{L_{H}^{2}+X_{S}^{2}}-L_{H}\approx \frac{1}{2}\frac{X_{S}^{2}}{L_{H}}. \end{array}$$

Therefore, the phase lag is represented by

(8) $$\begin{array}{c} \phi_{S}=k\cdot \text{MN}=\frac{\pi }{\lambda }\cdot \frac{X_{S}^{2}}{L_{H}}. \end{array}$$

Substituting the expression of the electric field intensity into the H-plane of the horn, we attain

(9) $$\begin{array}{c} \left.\begin{array}{c} E_{y}=E_{0}\cos\left(\frac{\pi X_{s}}{D_{1}}\right)e^{-j\left(\pi /\lambda \right)\left(X_{s}^{2}/L_{H}\right)}\\ H_{x}=-\frac{E_{y}}{120\pi } \end{array}\right\}. \end{array}$$

For the internal field distribution of the E-plane sector horn, the aperture field of the E-plane horn can be obtained by the same method by analyzing the H-plane horn expressed by

(10) $$\begin{array}{c} \left.\begin{array}{c} E_{y}=E_{0}\cos\left(\frac{\pi X_{s}}{D_{1}}\right)e^{-j\left(\pi /\lambda \right)\left(Y_{s}^{2}/L_{E}\right)}\\ H_{x}=-\frac{E_{y}}{120\pi } \end{array}\right\}. \end{array}$$

Currently, the amplitude distribution law of the aperture field is the same as that of the H-plane horn. Under the excitation of the TE_10_ wave, it is distributed in cosine form along the *X* direction and evenly along the *Y* direction. The phase of the aperture is different, and there is also a phase difference that, however, occurs in the *Y* direction.

The relationship between *D*_1_ and *D* is expressed by

(11) $$\begin{array}{c} \frac{D_{1}}{\sin\alpha }=\frac{D}{\sin\left(\pi -\left(\pi -\beta /2\right)\right)}, \end{array}$$

Namely, *D*_1_ = *D*(sin*α*/(sin(*β*/2))).

The amplitude of the aperture field of the pyramid horn can be considered the same as that of the fan-shaped horn on the H-plane and distributed according to the cosine form. On the E-plane, it can be considered the same as the fan-shaped horn. According to the uniform distribution, the phase of the aperture field is distributed (*π*/*λ*)((*X*_*S*_^2^/*L*_*H*_) + (*Y*_*S*_^2^/*L*_*E*_)). Therefore, the aperture field of the pyramid horn can be expressed by

(12) $$\begin{array}{c} E=E_{0}\cos\left(\frac{{\pi X}_{s}\sin\left(\beta /2\right)}{D\sin\alpha }\right)e^{-j\left(\pi /\lambda \right)\left(\left({X_{s}}^{2}/L_{H}\right)+\left({Y_{s}}^{2}/L_{E}\right)\right)}, \end{array}$$

where both *L*_*H*_ and *L*_*E*_ are the heights of the H-plane and E-plane of the constructed pyramid horn, respectively.

## 3. The Mathematical Model of the Temperature Field for the Microwave Heating

In this research, the discrete element method [20] was adopted. Asphalt is assumed to be heated as an isotropic material. Utilizing the conduction analysis of an infinitesimally small (differential) control volume (DCV) [21], *dx* · *dy* · *dz* in the asphalt pavement is shown in Figure 4 [22].

Equation (13) is obtained from the law of the conservation of energy.

(13) $$\begin{array}{c} {\dot{E}}_{\text{in}}+{\dot{E}}_{g}-{\dot{E}}_{\text{out}}={\dot{E}}_{\text{st}}, \end{array}$$

where ${\dot{E}}_{\text{in}}$ denotes the rate of the energy transfer into a control volume, ${\dot{E}}_{\text{out}}$ denotes the rate of the energy transfer out of a control volume, ${\dot{E}}_{\text{st}}$ represents the rate of the energy change in a control volume, *q* denotes heat transfer rate, *ρ* is its density, *c* is its specific heat capacity, *T* denotes temperature, *t* is time, and *x*, *y*, and *z* are rectangular coordinates, respectively. Thus,

(14) $$\begin{array}{c} {\dot{E}}_{g}=\dot{q}dxdydz, \end{array}$$

(15) $$\begin{array}{c} {\dot{E}}_{st}=\rho c\frac{\partial T}{\partial t}dxdydz, \end{array}$$

(16) $$\begin{array}{c} {\dot{E}}_{\text{in}}-{\dot{\;E}}_{\text{out}}=\frac{\partial q_{x}}{\partial x}dx+\frac{\partial q_{y}}{\partial y}dy+\frac{\partial q_{z}}{\partial z}dz, \end{array}$$

(17) $$\begin{array}{c} q_{x}=-k\frac{\partial T}{\partial x}dydz, \end{array}$$

(18) $$\begin{array}{c} q_{y}=-k\frac{\partial T}{\partial y}dxdz, \end{array}$$

(19) $$\begin{array}{c} q_{z}=-k\frac{\partial T}{\partial z}dxdy. \end{array}$$

Substituting Equations (14) through (19) simultaneously into Equation (13), it leads to the heat diffusion equation denoted by

(20) $$\begin{array}{c} k\left(\frac{\partial^{2}T}{\partial x^{2}}+\frac{\partial^{2}T}{\partial y^{2}}+\frac{\partial^{2}T}{\partial z^{2}}\right)+\dot{q}=\rho c\frac{\partial T}{\partial t}. \end{array}$$

In the process of a microwave heating asphalt mixture, if the internal heat source is the microwave power per unit volume, then the expression is defined by

(21) $$\begin{array}{c} \left(\frac{\partial^{2}T}{\partial x^{2}}+\frac{\partial^{2}T}{\partial y^{2}}+\frac{\partial^{2}T}{\partial z^{2}}\right)+P^{*}, \end{array}$$

(22) $$\begin{array}{c} k\left(\frac{\partial^{2}T}{\partial x^{2}}+\frac{\partial^{2}T}{\partial y^{2}}+\frac{\partial^{2}T}{\partial z^{2}}\right)+P^{*}=\rho c\frac{\partial T}{\partial t}. \end{array}$$

Besides, Equations (21) and (22) denote the temperature field model of a microwave-heated asphalt mixture. Thus, *P*∗ is represented by Equation (23) and *P*_*d*_ is represented by Equation (24).

(23) $$\begin{array}{c} P^{*}=\frac{\partial P\left(z\right)}{\partial z}=-\alpha P_{0}e^{-\alpha z}, \end{array}$$

(24) $$\begin{array}{c} P_{d}=\pi f\varepsilon_{0}\varepsilon^{\prime }tg\delta E^{2}. \end{array}$$

*E* denotes the distribution of the calculated aperture field.

## 4. The Results and Discussion

### 4.1. Simulation

The simulation model of a microwave heating asphalt mixture is established, as shown in Figure 5. Firstly, the microwave field is simulated in the Microwave Studio of the CST software. The simulation parameters are set as follows: the size of the horn antenna aperture is 120 × 90 mm, the relative dielectric constant of asphalt mixture is 8.5, the tangent of loss angle is 0.03, the specific heat capacity is 0.9 kJ/kg °C, the thermal conductivity is 0.55 W/k · m, and the density is 2020 kg/m^3^. Then, the data are imported into multiple physical fields to calculate the temperature field. The simulation parameters are microwave output power of 1.3 kW, the initial temperature of 10°C, and heating time of 14 min.

### 4.2. Experiment

The experimental scheme is defined as follows: the experimental devices are shown in Figure 6. To reduce the influence of many temperatures measuring thermocouples in an asphalt mixture on the distribution of the microwave field, five thermocouples were buried at the depths of Z = 3 cm, 6 cm, 9 cm, 12 cm, and 15 cm in the center of the material box. The temperature measuring points are shown in Figure 7. The temperatures of the different coordinates were measured by moving the horn antenna. After measuring the temperature field of one point, the asphalt mixture needs to be cooled down to room temperature, and then, a measurement is taken at another point. The coordinates of the temperature measuring points are as follows: (-50,-60), (-50,-30), (-50,0), (-50,30), and (-50,60); (-25,-60), (-25,-30), (-25,0), (-25,30), and (-25,60); (0,-60), (0,-30), (0,0), (0,30), (0,60); (25,-60), (25,-30), (25,0), (25,30), and (25,60); and (50,-60), (50,-30), (50,0), (50,30), and (50,60).

Maintaining and constructing asphalt pavements sustainably could be realized by microwave heating which is an auspicious method since it requires a minimum level of outside intervention. Some of the underlined issues are called overheating and nonuniform heating. Thus, both frequency and power are two attributes that are under investigation.

### 4.3. Discussion

Both Figure 8 and Table 1 depict the temperature field at the same depth *z* that is symmetrical about the *y* = 0 planes. Therefore, the experiment can be simplified further. At the same depth, 25 temperature measurement points in the experimental scheme can be simplified to 15 temperature measurement points: (-50,-60), (-50,-30), and (-50,0); (-25,-60), (-25,-30), and (-25,0); (0,-60), (0,-30), and (0,0); (25,-60), (25,-30), and (25,0); and (50,-60), (50,-30), and (50,0).

As shown in Figure 9, in the *y* = 0 and *y* = 30 planes, the simulation values tally with the experimental values highly. In the *y* = 60 plane, the simulation values tally with the experimental values relatively. The experimental area is located at the edge of the horn antenna and belongs to the low-temperature areas heated by the microwave sidelobe. The experimental values are slightly different from the simulation values. The reasons may be (1) the asphalt mixture used in the experiment cannot be completely uniform, (2) the processing error of the horn antenna leads to the change of the microwave field distribution, and (3) the opening surface of the horn antenna is not parallel to the asphalt mixture surface.

## 5. Conclusion

The aperture field of an oblique horn antenna is different from that of a straight horn antenna. The main reason is that the oblique horn antenna has an asymmetric structure, and there is an included angle between the microwave propagation direction and the aperture, while the microwave propagation direction of the straight horn antenna is vertical and the aperture outward.

The distribution of the temperature field of an oblique horn antenna is different from that of a straight horn antenna. At different depths of asphalt mixture, the highest point of the temperature field of the oblique horn antenna is not directly below the center of the horn surface, and it becomes closer and closer to the oblique edge with the increase of depth *z*. At different depths, the highest point of the temperature field of the straight horn antenna is directly below the center of the horn surface.

On the other hand, there is no one-to-one correspondence between the experimental outcomes and the simulation results. The potential difference could stem from those issues as follows: (1) the asphalt mixture used in the experiment cannot be completely uniform, (2) the processing error of the horn antenna leads to the change of the microwave field distribution, and (3) the opening surface of the horn antenna is not parallel to the asphalt mixture surface.

The horn antenna has symmetry, and the temperature field also has symmetry too. When measuring the temperature field, the measuring points can be reduced according to the actual situation to improve efficiency.

Consequently, the model owns high precision and can be used to guide the design of microwave heating equipment.

## Figures and Tables

**Figure 1:** The two kinds of the horn antennas. (a) A straight horn antenna. (b) An oblique horn antenna.

**Figure 2:** An oblique horn antenna.

**Figure 3:** The position relation of the horn caliber.

**Figure 4:** The energy flow of the microelement.

**Figure 5:** The simulation model.

**Figure 6:** A microwave heating unit.

**Figure 7:** The location of the temperature measuring points.

**Figure 8:** The distribution of the plane temperature when *x* = 0.

**Figure 9:** The plane temperature field when *Y* is set to different values. (a) The plane temperature field when *Y* = 0. (b) The temperature field when *Y* = 30. (c) The plane temperature field when *Y* = 60.

**Table 1:** The results of both simulation and computation.

*z* *y*	Simulation results					Calculation results				
	30	60	90	120	150	30	60	90	120	150
-60	34.9	31.2	28.1	25.5	23.2	36.9	31	30.1	19.1	20.7
-30	82.4	70.6	57.1	44.9	35.4	80.9	72.6	54.5	46	34.6
0	122.9	100.9	76.1	55.9	41.7	128.3	100.9	74.7	54.9	39.9
30	82.4	70.6	57.1	44.9	35.4	80.6	66.8	52.5	45.3	34.2
60	34.9	31.2	28.1	25.5	23.2	36	29.9	29.4	21.5	20.3

## Data Availability

Data will be provided upon request to the authors.
